This article has been retracted.

# miR-223-3p Regulates NLRP3 to Inhibit Proliferation and Promote Apoptosis of ONG Cells

**DOI:** 10.1155/2022/2805645

**Published:** 2022-10-04

**Authors:** Lili Nie, Hui Zou, Chi Ma, Xiaoke Wang

**Affiliations:** ^1^Department of Ophthalmology, The Second Hospital of Jilin University, Changchun, 130000 Jilin, China; ^2^Department of Neurosurgery, The First Hospital of Jilin University, Changchun, 130021 Jilin, China; ^3^Department of Neurosurgery, The Second Hospital of Jilin University, Changchun, 130000 Jilin, China

## Abstract

**Objective:**

Optic nerve glioma (ONG) is a rare disease, defined as a WHO grade I tumor, which affects the visual pathway. The objective of this study was to investigate the expression of miR-223-3p in ONG as well as its function and regulation in ONG cell lines.

**Methods:**

qRT-PCR assays were used to measure miR-223-3p expression in ONG tissues and cell lines. After overexpression of miR-223-3p in Hs683 and WERI-Rb-1 cell lines, CCK-8 and EdU assays were performed to examine cell proliferation, and flow cytometry was used to assess apoptosis. Dual luciferase assays were utilized to identify the target binding to miR-223-3p and NLRP3. Rescue assays were carried out to investigate the regulatory mechanism of miR-223-3p acting through NLRP3. Nude mouse tumorigenesis assays were established to verify the effect of miR-223-3p on ONG growth.

**Results:**

miR-223-3p was weakly expressed in both ONG tissues and cell lines. miR-223-3p inhibited the proliferative ability of Hs683 and WERI-Rb-1 cell lines and promoted apoptosis. In addition, there was binding between miR-223-3p and NLRP3. Simultaneous overexpression of NLRP3 and miR-223-3p partially counteracted the role of miR-223-3p in the cell lines. Lastly, miR-223-3p inhibited ONG growth.

**Conclusion:**

miR-223-3p plays an inhibitory role in ONG development by regulating NLRP3 to inhibit the proliferation of ONG cells and promote apoptosis.

## 1. Introduction

The role of the optic pathway is to transmit visual information from photoreceptors in the retina to the visual cortex in the brain. A variety of tumors involve the optic pathway, the most common of which is optic pathway glioma (OPG) [1]. OPG accounts for approximately 3% to 5% of CNS tumors in children and usually occurs in the first and second decades of life [1, 2]. The lesions grow along the optic pathway, from the optic nerve to the occipital cortex, including the optic cross and hypothalamic regions [3].

Optic nerve gliomas (ONG), classified as a type of OPG, are benign tumors classified as hairy cell astrocytomas. ONG may be associated with neurofibromatosis type 1 (NF-1) or may be disseminated [4]. OPG occurs in 15 to 20% of children with NF1, with some patients being asymptomatic and some presenting symptoms such as vision loss. Children diagnosed with ONG will experience some visual loss, with a higher risk of visual loss in sporadic ONG compared to ONG secondary to NF1 [5]. ONG most often presents as WHO grade I hairy cell astrocytoma, is diagnosed in childhood, and mostly conforms to a benign clinical course, whereas the rarer malignant ONG (WHO grades III–IV) is more common in adults and more aggressive with rapid vision loss and death within a few months [6, 7].

The diagnosis of ONG is usually based on neuroimaging and a comprehensive clinical examination, but the variable clinical growth pattern of ONG and the lack of standardized measurements lead to variable outcomes after treatment. Current treatments for ONG include standard chemotherapy, molecular targeted therapy, radiation therapy, and surgery. Given the many known side effects of chemotherapy and radiotherapy, chemotherapy is prone to induce secondary leukemia, among other types of cancer, and radiotherapy associates with a range of complications. The risk of vision loss is high if surgery is performed. On the other hand, molecular targeted therapy has achieved remarkable clinical success in treatment. Research related to molecular targeted therapy for ONG disease can help to further understand the molecular mechanisms of disease and therapeutic prospects of ONG.

MicroRNAs (miRNAs) are a class of highly conserved tissue-specific, small non-protein-coding RNAs that maintain cellular homeostasis through negative gene regulation [8]. miRNAs affect gene expression mainly by targeting mRNAs. Any change in miRNA expression may affect the degree of target regulation and, thus, cellular homeostasis [9]. Abnormally expressed miRNAs are associated with cancer cell behavior and can serve as potential markers and therapeutic targets, and due to specific and stable expression, miRNAs have led to new directions for cancer therapy [10, 11].

There are few studies on the association between miRNAs and ONG. Only a few studies have addressed the association of miRNAs with glioma. For example, increased expression of circCCDC66 in glioma promotes tumor development and metastasis through miR-320a-mediated regulation of FOXM1 expression [12]. Studies have shown that miR-223-3p acts as a novel microRNA regulator in the biological behavior of various types of tumor cells. miR-223-3p regulates hepatocarcinogenesis by targeting the FAT1 gene [13]. Knockdown of miR-223-3p can inhibit the progression of NSCLC cells by targeting RHOB [14]. In this study, we investigated the role of miR-223-3p in ONG cells.

## 2. Materials and Methods

### 2.1. Sample Collection

Clinical samples were collected from seven patients treated surgically at our hospital for ONG between October 2019 and July 2020. ONG tissues and paired paraneoplastic nontumor tissues were collected during surgery. ONG tissue collection avoided the collection of necrotic tissues. Paraneoplastic nontumor tissues were selected at a distance of 2 cm or more from the tumor, and the specimens were marked accordingly and placed in a liquid nitrogen tank for rapid cooling and subsequent storage. All specimens were collected within 30 min of surgical excision. The inclusion and exclusion criteria for cases are as follows: Patients under 70 years of age, undergoing surgery only, and not receiving preoperative chemotherapy or radiation therapy; pathologically diagnosed with definite optic glioma; and no any other type of cancer, autoimmune disease, infectious disease, etc.

### 2.2. Cell Culture and Transfection

The medium for the Hs683 cell line (ATCC) was DMEM supplemented with 10% FBS, and the medium for the WERI-Rb-1 cell line (National Collection of Authenticated Cell Cultures) was RPMI-1640 supplemented with 10% FBS. The cells were incubated at 37°C in a 5% CO_2_ saturated humidity incubator, and the cells were passaged when the confluence reached 70%. The cell transfection procedure was performed according to the instructions of Lipofectamine 2000 reagent. The specific steps are as follows. 1 d before transfection, we performed digestion with trypsin, harvested cells grown in log phase, counted them, and inoculated them into the corresponding culture dishes. Transfection was performed by incubating overnight until the cell growth density reached 50%, and the medium was changed to a new one 1 h before transfection. We used Lipofectamine 2000 reagent for transfection. In a 12-well plate, for example, 100 *μ*L of saline without serum and antibiotics was added to each of two sterile 1.5 mL centrifuge tubes, and plasmid DNA or miRNA was added to one of them, and the liposome transfection reagent was added to the other. Mix individually and leave at room temperature for 5 min, then mix the two tubes drop by drop and leave at room temperature for 20 min. Add the mixture drop by drop to the culture solution, mix gently, and incubate at 37°C and 5% CO_2_ incubator, and change the solution once around 6 h. Finally, the culture medium was changed and the cells were collected after 48 h.

### 2.3. Detection of Cell Proliferation by CCK-8 Assay

ONG cells were cultured until the logarithmic growth phase of the cells, and the cells were digested using trypsin and the cell suspensions were collected. The cell suspension was centrifuged and separated to obtain cell precipitate, which was then resuspended in the culture medium and the number of cells was counted. The cell suspension was then inoculated into a 6-well culture plate, and transfection was performed after the cells had grown to 50% of the well area. After 48 hours of transfection operation, ONG cells were digested with trypsin, the cell suspension was collected, centrifuged, resuspended, and counted and subsequently inoculated in 96-well culture plates (1500 cells per well). Six replicate wells were set up for culture at each assay time point, and the total volume of medium in each well reached the level of 100 *μ*L. The ONG cells inoculated above were incubated continuously in a saturated humidity cell culture incubator at 37°C and 5% CO_2_, and CCK-8 detection reagent (10 *μ*L per well) was added at the 0th and 48th hours of culture, respectively, and incubated in the cell culture incubator for 3 hours before detection. The absorbance value at wavelength 450 nm (OD450) was measured by enzyme-linked immunoassay.

### 2.4. Gene Expression Detection by qRT-PCR

(1) Sample preparation: for clinical tissue samples, the samples were removed from the liquid nitrogen tank, trimmed to about 5 mm diameter tissue mass, rinsed 2-3 times with DEPC water, crushed by ultrasonic crusher, added 1 mL TRIzol solution, blown and mixed, and placed in an ice box for 10 min to make full contact between lysate and tissue. For cell samples, remove the cells from the incubator, discard the medium, wash 2-3 times with PBS, add 1 mL TRIzol lysis solution, scrape off the cells, transfer them to 1.5 mL EP tubes, repeatedly blow and mix, and set aside in an ice box for 10 min. (2) RNA extraction: add 0.2 mL of chloroform to the well-mixed cell/tissue TRIzol mixture, shake vigorously for 15 s to make it well mixed, and leave it for 10 min at room temperature. Centrifuge at 12000 g/min for 10 min at 4°C and remove. After centrifugation, the liquid was divided into three layers, the upper layer was the colorless aqueous phase, the lower layer was the organic phase, and the middle layer was the cell debris layer. Carefully aspirate the upper aqueous layer into a new EP tube, avoiding touching the middle cell debris layer. After that, add the same amount of isopropanol as the upper aqueous layer to precipitate RNA, mix thoroughly, and leave it at room temperature for 10 minutes. After that, continue to centrifuge at 4°C at 12000 g/min for 10 minutes and observe the white precipitation of RNA in the EP tube, after discarding the supernatant. Wash the white precipitate with 0.2 mL of 75% ethanol, centrifuge at 12000 g/min for 5 min at 4°C, and repeat twice. Discard the supernatant after washing and dry at room temperature for 30 min, taking care to avoid overdrying. After that, add 20-30 *μ*L of water without RNAse to dissolve the RNA. (3) Total RNA was reverse transcribed into cDNA using the RevertAid First-Strand cDNA Synthesis kit. qRT-PCR analysis was performed using the SYBR Premix Ex Taq II Kit in an ABI PRISM 7300 sequence detection system. The 2^-*ΔΔ*Ct^ method was used to calculate the expression levels of miR-223-3p and NLRP3, followed by normalization against the expression levels of U6 and GAPDH, respectively. The primer sequences of miR-223-3p is F: 5′-ACACTCCAGCTGGGTGTCAGTTTGTCAAAT-3′ and R: 5′-CTCAACTGGTGTCGTGGAGTCGGCAATTCAGTTGAGTGGGGTAT-3′ [15] and the primer sequences of NLRP3 is F: 5′-AAAAGACTCATCCGTGTGCC-3′ and R: 5'-TTCCTGGCATATCACAGTGG-3′ [16]

### 2.5. EdU Assay

(1) EdU labeling of cultured cells and fixation, washing, and permeabilization: first, we prepared 2× of EdU working solution. Since EdU working solution is added to the well plate in equal volume with the culture medium, we need to prepare a 2× working solution using a final concentration of 10 *μ*M (1×) of EdU. Specifically, a 2× EdU working solution (20 *μ*M) can be obtained by diluting EdU (10 mM) 1 : 500 with the cell culture medium. Add an equal volume of the 2× EdU working solution (20 *μ*M) prewarmed at 37°C to a 6-well plate to make the final concentration of EdU in the 6-well plate 1×. Continue to incubate the cells for 2 hours. Next, after EdU-labeled cells were completed, the culture medium was removed and 1 mL of fixative was added and fixed at room temperature for 15 minutes. Then, remove the fixative and wash the cells with 1 mL of washing solution 3 times per well for 3-5 minutes each time. Remove the washing solution and incubate with 1 mL of permeabilizing solution per well for 10-15 minutes at room temperature. Further, the permeabilizing solution was removed and the cells were washed 1-2 times per well with 1 mL of washing solution for 3-5 minutes each time. (2) EdU detection: first, prepare the click additive solution. In detail, dissolve one tube of click additive with 1.3 mL of deionized water and mix until all dissolved, that is, click additive solution. Then, prepare the click reaction solution. In the next step, remove the washing solution from the previous step. Then, add 0.5 mL click reaction solution to each well and gently shake the plate to ensure that the reaction mixture can cover the sample evenly. Incubate for 30 minutes at room temperature and protected from light. Next, the click reaction solution is aspirated and washed 3 times with washing solution for 3-5 minutes each. Finally, we use flow cytometry to perform the assay

### 2.6. Flow Cytometry Assay for Apoptosis

Briefly, each group of cells was first labeled with propidium iodide (PI)/Annexin-V (membrane-linked protein), and then, the number of apoptotic cells was detected by flow cytometry (Thermo Fisher Scientific Inc., Waltham, MA, USA). Specifically, the medium in each well of the culture plate was first aspirated, and the cells were carefully washed with PBS and kept on ice. Cells were separated using trypsin and resuspended, and the isolated cells were added dropwise to the diluent for further examination. Next, 1.0 × 10^6^ cells were mixed with 10 mL of binding buffer and 1.25 mL of Annexin V-Fluorescein Isothiocyanate in a dark room and incubated for 15 min at room temperature in a dark box. The cell suspension was centrifuged at 1000 g for 5 min, the supernatant was discarded, and 0.5 mL of ice-cold 1× binding buffer was added for resuspension. Finally, cells were incubated with 10 mL PI and transferred to fluorescence-activated cell sorting tubes (Fahrenheit, Munich, Germ any). Fluorescence signals were collected by flow cytometry.

### 2.7. Statistical Methods

Statistical analysis was performed using SPSS 21.0 software (SPSS, Chicago, IL, USA). Results were expressed as mean ± standard deviation (SD). One-way or two-way analysis of variance (ANOVA) after Tukey's post hoc test was used to show the differences between experimental groups. *P* < 0.05 was statistically significant.

## 3. Results

### 3.1. miR-223-3p Is Weakly Expressed in ONG

The results of qRT-PCR assays showed that miR-223-3p was weakly expressed in ONG tissues compared with normal tissues (Figure 1(a)), and miR-223-3p was weakly expressed in the Hs683 and WERI-Rb-1 cell lines compared with the retinal epithelial cell line APRE-19 (Figure 1(b)).

### 3.2. miR-223-3p Exerts Oncogenic Effects in ONG Cell Lines

After successful overexpression of miR-223-3p in the Hs683 and WERI-Rb-1 cell lines (Figure 2(a)), we examined the changes in the cell proliferative ability by CCK-8 and EdU assays, and the results showed that miR-223-3p inhibited cell proliferation (Figures 2(b) and 2(c)). The flow cytometric results showed that miR-223-3p promoted apoptosis (Figure 2(d)).

### 3.3. miR-223-3p Directly Binds to NLRP3

It has been reported that miR-223-3p binds to NLRP3 in endothelial cells [17]. We verified this in the ONG cell lines by a dual luciferase assay (Figure 3(a)). qRT-PCR assays were used to detect the NLRP3 level in ONG tissues, and the results showed that NLRP3 was highly expressed in ONG tissues (Figure 3(b)). Moreover, the level of NLRP3 decreased under miR-223-3p overexpression (Figure 3(c)).

### 3.4. miR-223-3p Regulates NLRP3

To investigate the involvement of NLRP3 in the miR-223-3p-related pathway, we overexpressed NLRP3 simultaneously in ONG cell lines overexpressing miR-223-3p. The results showed that overexpression of NLRP3 could partially counteract the decrease in proliferation (Figures 4(a) and 4(b)) and the increase in apoptosis (Figure 4(c)) of ONG cells caused by miR-223-3p. These findings indicate that miR-223-3p regulates NLRP3.

### 3.5. miR-223-3p Inhibits the Tumorigenic Ability of ONG Cells *In Vivo*

We examined the effect of miR-223-3p on the *in vivo* tumorigenic ability of ONG cells by tumorigenic assays in nude mice. The results showed that miR-223-3p inhibited the tumorigenic ability of WERI-Rb-1 cells in nude mice by yielding tumors with relatively lower weights (Figure 5(a)). In the isolated tumors, miR-223-3p expression was higher in the miR-223-3p group than in the control group (Figure 5(b)).

## 4. Discussion

ONG, a rare disease that is usually slow growing, is classified as a WHO grade I tumor that affects visual pathways. ONG is most common in children and is mostly benign, but malignant ONG also occurs in adults and has a more aggressive and fatal clinical presentation. ONG is a component of OPG disease that is rare and difficult to manage. Clinical treatment can involve chemotherapy, radiotherapy, and surgical resection, but all are limited by several factors, such as the high 3-year progression-free survival after treatment with carboplatin and vincristine in patients with gliomas aged 5 years or younger and the low 3-year progression-free survival in older patients [18]. Radiotherapy patients have a high survival rate but associate with more adverse consequences, leading to endocrine abnormalities, cerebrovascular disease, visual impairment, secondary malignancies, and neurocognitive deficits, especially in young patients with developing brains [5]. Primary surgery does not appear to be significantly beneficial in children younger than 2 years of age or in tumors with mucinous-like features [19]. Considering the risks of these three treatment modalities, there is a need to investigate the intrinsic molecular mechanisms to find safer and more effective treatment approaches. It has been shown that aberrant expression of microRNAs is closely associated with glioma formation, making them potential new markers and therapeutic targets for the diagnosis and treatment of glioma-like diseases [20, 21]. This study explores the role played by miR-223-3p in ONG.

An increasing number of human studies have reported that miRNAs are involved in tumorigenesis as oncogenes or tumor suppressors [23–25]. The identification of specific miRNAs in cancer cells is of great value for diagnostic and therapeutic intervention. There are few studies on ONG-related miRNAs, and most studies have focused on miRNAs involved in human gliomas. miR-223-3p has been shown to be associated with a variety of diseases, including cardiovascular diseases [26], prostate diseases [27], type 2 diabetes [28], and Parkinson's disease [29]. miR-223-3p can regulate downstream signaling pathways and play important roles in various tumors, and it is a potential therapeutic target. In the present study, we found that miR-223-3p was weakly expressed in ONG, and after successful overexpression of miR-223-3p in the Hs683 and WERI-Rb-1 cell lines, miR-223-3p inhibited cell proliferation and promoted apoptosis. Compared to normal cell lines, the miR-223-3p level was found to be highly expressed in neuroblastoma cell lines, and knockdown of miR-223-3p expression decreased cell growth and invasion but increased apoptosis [30]. miR-223-3p has been found to be upregulated in non-small-cell lung cancer tissues and cell lines, and high miR-223-3p expression resulted in poor patient survival [31]. miR-233-3p was weakly expressed in oral squamous cell carcinoma tissues and cells and exerted oncogenic effects by targeting SHOX2 [32]. These studies demonstrate the different mechanisms and roles of miR-223-3p in different tumors.

Our study further revealed that miR-223-3p binds to NLRP3 and may exert oncogenic effects by regulating NLRP3. The results of the present study showed that overexpression of NLRP3 could partially counteract the decrease in proliferation and the increase in apoptosis of ONG cells induced by miR-223-3p, indicating that miR-223-3p exercised its function in ONG cells by regulating NLRP3. NLRP3 is a target of miR-223-3p, and NLRP3 can be regulated by miR-223-3p in different physiological and pathological processes. In addition, miR-223-3p induces NLRP3 inflammasome inactivation in breast cancer, inhibits tumor growth, and enhances anticancer immunity [33]. miR-22-3p also plays an inhibitory role in retinal pigment epithelial damage by targeting NLRP3 [34]. The present study contains some limitations. Firstly, miR-223-3p has many potential target genes, and only one of them, NLRP3, was detected in this study. Secondly, we did not further elucidate the signaling pathways downstream of NLRP3 that may be regulated. And thirdly, this study further needs to validate the function of miR-223-3p in an in situ tumorigenic animal model.

## 5. Conclusion

We showed that miR-223-3p can promote apoptosis and inhibit ONG cell proliferation by regulating NLRP3, and miR-223-3p can be used as a biomarker for the treatment of ONG.

## Figures and Tables

**Figure 1:** Weak expression of miR-223-3p in ONG tissues and cell lines. qRT-PCR assays were used to detect the expression of miR-223-3p in ONG tissues (a) and cell lines (b).

**Figure 2:** Function of miR-223-3p in ONG cell lines. (a) qRT-PCR assays were used to detect the overexpression efficiency of miR-223-3p in ONG cell lines. (b) CCK-8 assays and (c) EdU assays were used to investigate the effect of miR-223-3p on the proliferation of ONG cell lines. (d) Flow cytometry was used to detect the effect of miR-223-3p on the survival of ONG cell lines.

**Figure 3:** NLRP3 directly binds to miR-223-3p. (a) Dual luciferase assays were used to verify the binding between miR-223-3p and NLRP3 3′-UTR region in the ONG cell lines. (b) qRT-PCR assay was used to detect the expression of NLRP3 in ONG tissues. (c) qRT-PCR assay was used to detect the expression of NLRP3 under miR-223-3p overexpression.

**Figure 4:** miR-223-3p regulates NLRP3. (a) CCK-8 assays and (b) EdU assays were performed to detect the effects of miR-223-3 and NLRP3 on the proliferation of ONG cell lines. (c) Flow cytometry was used to detect the effect of miR-223-3p and NLRP3 on the apoptosis of ONG cell lines.

**Figure 5:** miR-223-3p inhibits the tumorigenic ability of ONG cells *in vivo*. (a) The effect of miR-223-3p on the *in vivo* tumorigenic ability of ONG cells was measured by the weights of the harvested tumors in nude mice tumorigenic assays. (b) qRT-PCR assay was used to detect the expression of miR-223-3p in tumors.

## Data Availability

No data were used to support this study.
